RETRACTED

# The biofilm formation and antibiotic resistance of bacterial profile from endotracheal tube of patients admitted to intensive care unit in southwest of Iran

**DOI:** 10.1371/journal.pone.0277329

**Published:** 2022-11-17

**Authors:** Zahra Dargahi, Anas Abdullah Hamad, Ahmad Farajzade Sheikh, Nazanin Ahmad Khosravi, Shahla Samei Fard, Moloudsadat Motahar, Fatemeh Jahangiri Mehr, Fariba Abbasi, Hossein Meghdadi, Pejman Bakhtiyariniya, Reza Heydari, Melika Moradi, Aram Asareh Zadegan Dezfuli

**Affiliations:** 1 Student Research Committee, Ahvaz Jundishapur University of Medical Sciences, Ahvaz, Iran; 2 Department of Microbiology, Faculty of Medicine, Ahvaz Jundishapur University of Medical Sciences, Ahvaz, Iran; 3 Department of Medical Laboratory Techniques, Al Maarif University College, Al Anbar, Ramadi, Iraq; 4 Infectious and Tropical Diseases Research Center, Health Research Institute, Ahvaz Jundishapur University of Medical Sciences, Ahvaz, Iran; 5 Pain Research Center, Health Research Institute, Ahvaz Jundishapur University of Medical Sciences, Ahvaz, Iran; 6 Department of Microbiology, Golestan Hospital, Ahvaz Jundishapur University of Medical Sciences, Ahvaz, Iran; Qassim University, College of Public Health and Informatics, SAUDI ARABIA

## Abstract

Ventilator-associated pneumonia (VAP) is a prevalent nosocomial illness in mechanically ventilated patients. Hence, the aim of this study was to investigate the pattern of antibiotic resistance and biofilm formation of bacterial profiles from Endotracheal Tubes of patients hospitalized in an intensive care unit in southwest Iran. According to the standard operating method, the microbiological laboratory conducts bacteria culture and susceptibility testing on endotracheal Tube samples suspected of carrying a bacterial infection. The Clinical and laboratory standards institute (CLSI) techniques are used to determine the Antimicrobial resistance (AMR) of bacterial isolates to antibiotics using the disk diffusion method. The crystal violet staining method was used to assess the biofilm-forming potential of isolates in a 96-well microtiter plate. In total, (51%) GPBs were included in this study. The isolated GPB were coagulase-negative Staphylococcus (16%), S. aureus (14%). In total, (40%) of GNB were included in this study. The isolated GNB were Klebsiella spp. (36%), A. baumannii (22%), P. aeruginosa (35%). (32%) bacterial strains were MDR and (29%) strains were XDR. The results of biofilm formation showed (72%) were biofilm producers. VAP is a common and severe nosocomial infection in mechanically ventilated patients. Controlling biofilm formation, whether on the ET or in the oropharyngeal cavity, is thus an important technique for treating VAP. Colistin and linezolid are antibiotics that are effective against practically all resistant GNB and GPB isolates.

RETRACTED

## Introduction

Ventilator-associated pneumonia (VAP) is known as a prevalent and deadly nosocomial infection in mechanically ventilated patients, mostly resulting in high mortality, and also long-term intensive care unit (ICU), longer duration of hospitalization, and increased cost. Over the last decades, the role of the endotracheal tube (ET) in VAP pathogenesis and also medical device-related infections has become prominent [1]. VAP is pneumonia that develops within 48–72 after endotracheal intubation and mechanical ventilation. Patients who suffer from this infection may present with a new or continuous infiltrate on chest radiography, together with fever, increased leukocyte count, and alterations in sputum features. Early VAP happens within the first 2–4 days of ventilation and is often caused by bacteria that are sensitive to antibiotics. Early VAP, on the other hand, occurs after 4 days and appears to be produced by multidrug-resistant bacteria [2]. Due to the presence of various infections caused by hospital pathogens such as *Pseudomonas aeruginosa*, *Acinetobacter baumannii*, or methicillin-resistant *Staphylococcus aureus* (MRSA), the recognition of VAP from other infections is of high priority. Coagulase-negative staphylococcus (CoNS) has been indicated to be resistant to some or all antibiotics, and the resultant infections mostly result in mortality in 13–25.5% of patients [3–5]. It is notable that in the ICU, 50% of the antibiotics recommended are for VAP management [6]. In the absence of a standard approach for VAP management, it is estimated that by 2050, approximately 10 million people will die each year as a result of resistance to antibiotics [7].

In intubated patients, the biofilm formation on ET is an early and constant process, and ET behaves as a reservoir to infect microorganisms. Immediately after intubation, a mixed biofilm, with the ability to harbor microbial pathogens, is formed on the ET. Microorganisms can exist as individual cells in a liquid medium or as an immobile community in biofilms [8]. A microbial biofilm is a three-dimensional collection of microbial cells enclosed in a self-produced matrix that protects it from the harsh environment. The matrix-enclosed communities of bacteria stick to each other and are adherent to inert or living surfaces; as a result, in these protected populations, the hosted microorganisms are able to survive in a dormant state. These persister cells, which seem to be metabolically inactive, make up a minor portion of the biofilm and remain in an immobile condition due to a slowed metabolism because they’re less vulnerable to the effects of antimicrobials [9].

RETRACTED

A growing body of research shows that the incidence of antibiotic resistance varies geographically because there is some resistance to next-generation antibiotics. Such resistance appears to be an alarm, encouraging physicians to periodically examine the antibiotic resistance patterns and exploit these models for experimental and special treatment of infections [10–13]. Thus, each region needs to check dynamically and sustainably the patterns of its resistance and sensitivity so that the outcomes are applied as a guide for the appropriate administration of antibiotics in the aforesaid region. This action is of paramount importance in the ICU [14]. As a consequence, this study was carried out to assess the biofilm formation and antibiotic resistance of bacterial profile from Endotracheal Tube of patients admitted to Intensive care unit in the southwest Iran.

### Inclusion criteria

The inclusion criteria were over 18 years of age and at least 5-day survival after intubation. Patient information, including gender, age, positive culture of tracheal secretions, type of cultured microorganism, sensitivity, and resistance to tested antibiotics was recorded for each patient.

## Methods

### Study design

This cross-sectional study was conducted from June 2020 to June 2021. The investigation included all clinical samples sent to the Golestan Hospital microbiology laboratory in Ahvaz, Iran. The hospital serves as a referral center for the public hospital in Ahvaz city.

### Sample techniques and collection

The microbiological lab performed for bacteria were culture and sensitivity tests on the endotracheal Tube samples suspected of any bacterial infection based on the standard operating procedure. Specimens were obtained from ICU patients with a tracheal tube with endotracheal aspiration, when they had a clinical manifestation of pneumonia (cough, purulent respiratory secretion, fever & new or progressive infiltration of the lung in CXR) and were referred to the laboratory in the special sterile bottles (Lukens trap).

### Microbial identification

All samples are cultured on an appropriate culture media—i.e. blood culture is conducted whenever a blood-stream infection is expected, in trypticase soy broth prepared in the laboratory. If there is an indication of growth like hemolysis, gas, and turbidity, the inoculum would be subcultured on an appropriate solid medium for further identification. Non-fastidious bacteria would be cultivated on Blood and MacConkey agar, whereas fastidious bacteria would be grown on Chocolate agar. The single bacterial colony from culture media would be taken for Gram staining. For preliminary identification of the bacteria, Gram staining and colony features are used. Gram-positive bacteria (GPB) would be cultured in blood agar, and mannitol salt agar. for suspected enterococcal colonies, we used a bile esculin test identified using catalase, coagulase, bacitracin, pyrrolidinyl acrylamides (PYRase), optochin bile solubility, and Novobiocin. Gram-negative bacteria (GNB) would be cultured in MacConkey agar and Eosin methylene blue agar. Then identified based on serial biochemical reactions and fermentation of carbohydrates i.e. oxidase, catalase, triple sugar iron agar, citrate utilization test, urease, lysine iron agar, Sulphur indole motility, and indole test. Standard strains were used for all tests and suspicious tests were checked twice [15].

RETRACTED

### Antibiotic resistance AMR profiles

The AMR of bacterial isolates to antibiotics is evaluated using the disk diffusion method in accordance with CLSI standards (2022). The isolates are classified as sensitive and resistant based on the diameter of the clearing zone according to CLSI (2022) guidelines. The antibiotic discs represented: ciprofloxacin (Fluorinated quinolones), clindamycin (Lincosamides), gentamycin (Aminoglycosides), erythromycin (Macrolides), sulphamethoxazole/trimethoprim (Sulphonamides), tetracycline (Tetracyclines), vancomycin (Glycopeptides), Quinupristin-dalfopristin (streptogramins), cefoxitin (penicillinase-stable penicillins), nitrofurantoin (nitrofurantoin), rifampin (ansamycins), and linezolid (oxazolidinones).

For antimicrobial drug susceptibility assay in Gram-negative anaerobic bacteria isolated from these infections, the Minimum Inhibitory Concentration (MIC) of imipenem, chloramphenicol, metronidazole, clindamycin, cefoxitin, and penicillin G (Sigma Chemical Co. USA) was determined by the agar dilution method. MIC of penicillin, metronidazole, clindamycin, and cefoxitin for Gram-positive anaerobic bacteria were determined by Etest strip (AB biomerieux, Sweden) according to CLSI guidelines for anaerobic susceptibility testing. The phenotype is defined as multiple drug resistance (MDR), extremely drug-resistant (XDR), and pan-drug-resistant (PDR) according to the International Expert proposal for Interim Standards Guidelines [16, 17].

### Biofilm formation

The crystal violet staining method was used to assess the biofilm forming potential of isolates in a 96-well microtiter plate. First, these isolates were inoculated in Mueller–Hinton agar at 37°C overnight. Then, these isolates were adjusted to 0.5 McFarland (~1.5×10^8^ CFU/ mL) with normal saline (0.85% NaCl). A 10-μL aliquot of each suspension was then diluted 1:200 in 190 μL of tryptic soy broth (TSB) containing 1% glucose in 96-well polystyrene microtiter plates. Following incubation at 37°C overnight, the plates were washed three times with PBS, fixed by adding 200 μL of methanol into each well, and stained with 200 μL of 0.1% crystal violet (CV) for 20 minutes. The plates were rinsed three times further to eliminate excess stain, and the residual CV was solubilized by incubating in 200 L of 95% ethanol for 10 minutes. The optical density at 570 nm (OD570) of each well was measured by the ELISA plate reader (μQuant; BioTek Instruments, Winooski, VT, USA), to evaluate the biofilm formation capacity. *S*. *epidermidis* ATCC 35984 and TSB broth were used as positive and negative controls (ODc) for the biofilm formation, respectively. The results were interpreted according to the criteria suggested by Zhang et al. Briefly, the isolates were classified into the several groups about the biofilm formation capacity: OD570≤ODc = no biofilm producer; ODc<OD570≤2×ODc = weak biofilm producer; 2×ODc<OD570≤4×ODc = moderate biofilm producer; and 4×ODc<OD570 = strong biofilm producer [18]. All experiments were performed in triplicate.

RETRACTED

### Ethics statement

This study was approved by the Research Ethics Committee (REC) of the Ahvaz Jundishapur University of Medical Sciences (IR.AJUMS.REC.1399.38). Informed written consent was obtained from the patients or their relatives (for patients under the age of 18 years).

## Results

### Dissemination of positive cultures/specimens

During the period of study, 1139 bacterial positive growth samples were collected from patients. Most of the isolates were obtained from female patients and were detected in adults in the age range of 18–24 years (n = 470; 41%), followed by the age group of 24–64 years (n = 471; 41%). Duration of being intubated was evaluated; it was shown that duration of being intubated had a median of 9 days (Between 2 to 60 days). We were only focused in this investigation if there was an underlying illness. Underlying diseases are some diseases such as DM (diabetes mellitus), HTN (hypertension), hyperlipidemia, cardiovascular diseases, pulmonary diseases, and renal diseases. Patients over the age of 64 were found to have the fewest isolates. Table 1 shows the age and gender distribution of patients with bacterial isolates.

**Table 1:** Age and sex distribution of patients with bacterial isolates.

Age group (y)	Total		
Sex	Male	Female	Bacteria
	N (%)	N (%)	N (%)
18–24	102(32%)	368 (44%)	470 (41%)
24–64	121 (38%)	350 (55%)	471 (41%)
> 64	95 (29%)	100 (12%)	195 (17%)
Total	318 (27%)	818 (72%)	1136 (100)

### Number of Gram positive of bacterial (GPB) and (GBN) isolates from endotracheal tube cultures of patients

In total, 593 GPBs (51%) were included in this study. The isolated GPB were coagulase-negative Staphylococcus (CoNS; n = 100/590; 16%), *S*. *aureus* (n = 119/590; 14%), *Enterococcus* spp. (n = 32/590; 0.05%), *Streptococcus* spp. (n = 277/590; 46%) and *Corynebacterium* spp. (n = 62/590; 10%) (Table 2). This study includes a total of 546 GNB (40%) were included in this study. The isolated GNB were *Klebsiella* spp. (n = 197/546; 36%), *A*. *baumannii* (n = 121/546; 22%), *P*. *aeruginosa* (n = 195/546; 35%) and *Neisseria gonorrhoeae* (n = 33/546; 0.06%) (Table 3).

RETRACTED

**Table 2:** Antibiotic resistance pattern for Gram-positive bacteria.

Gram-negative microorganisms															
Antibiotics	*S*. *aureus*			*Enterococcus* spp.			*Corynebacterium*.spp			*Streptococcus* spp.			CoNS		
	(n = 119)			(n = 32)			(n = 62)			(n = 277)			(n = 100)		
	U	S	R	U	S	R	U	S	R	U	S	R	U	S	R
**AMK**	-	50	69	-	19	13	-	12	50	+	-	-	-	25	75
**AMP**	-	72	47	-	12	20	-	42	19	+	-	-	-	12	88
**CZO**	-	112	7	-	30	2	-	23	39	+	-	-	-	32	68
**FEP**	-	119	-	-	28	4	-	19	43	-	96	181	-	41	59
**CTX**	-	119	-	-	20	12	-	35	27	-	57	220	-	50	50
**FOX**	-	77	42	S	17	15	-	55	7	+	-	-	-	52	48
**CRO**	+	-	-	+	-	-	+	-	-	+	-	-	+	-	-
**CIP**	-	66	53	-	9	23	-	32	30	+	-	-	-	42	58
**CLI**	-	67	52	-	8	24	-	12	50	-	112	165	-	58	42
**DOX**	-	74	45	-	23	10	-	31	31	+	-	-	-	52	48
**ERY**	-	59	60	-	4	28	-	41	21	-	213	64	-	22	78
**GEN**	-	84	35	-	21	11	-	22	40	+	-	-	-	31	69
**IMP**	+	-	-	+	+	+	+	-	-	-	115	162	-	19	81
**NIT**	-	97	22	-	32	-	-	32	30	+	-	-	-	31	69
**PEN**	-	55	64	-	-	32	-	30	32	-	51	226	-	42	58
**TZP**	-	107	12	-	20	12	-	41	21	+	-	-	-	74	26
**RIF**	-	73	46	-	24	8	-	51	11	-	200	77	-	61	39
**TCY**	-	99	20	-	18	14	-	34	28	-	87	190	-	62	39
**SXT**	-	66	53	-	23	10	-	32	30	-	225	52	-	63	37
**VAN**	-	109	10	-	10	22	+	-	-	-	74	203	-	60	40
**BAC**	-	-	117	-	-	32	+	-	-	+	-	-	-	62	38
**CAZ**	-	107	12	-	27	5	-	28	34	+	-	-	-	72	28
**SAM**	-	95	24	-	23	9	-	50	12	+	-	-	-	58	42
**TEC**	-	86	33	-	32	-	-	32	30	+	-	-	-	89	11
**LEV**	-	75	44	-	21	11	-	25	37	-	112	165	-	1S	85
**MUP**	-	88	31	_	23	10	+	-	-	+	-	-	-	72	28
**MNO**	-	99	20	_	20	12	-	26	36	+	-	-	-	59	41
**LNZ**	-	114	5	-	31	1	-	62	-	-	277	-	-	100	-
**COL**	+	-	-	+	-	-	+	-	-	+	-	-	+	-	-
**CCV**	-	97	22	+	-	-	-	23	39	+	-	-	-	64	36

Ampicillin (AMP), Gentamicin (GEN), Ciprofloxacin (CIP), Vancomycin (VAN), Ceftazidime (CAZ), Nitrofurantoin (NIT), Imipenem (IMI), Penicillin (PEN), Clindamycin (CLI), Erythromycin (ERY), Doxycycline (DOX), Trimethoprim/sulfamethoxazole (SXT), Colistin (COL), Linezolid (LNZ), Mupirocin (MUP), Rifampin (RIF), Amikacin (AMK), Ceftriaxone (CRO), Ceftazidime/Clavulanic acid (CCV), Minocycline (MNO), Cefazolin (CZO), Piperacillin/Tazobactam (TZP), Tetracycline (TCY), Ampicillin/Sulbactam (SAM), Teicoplanin (TEC), Levofloxacin, (LEV), Bacitracin (BAC), Cefoxitin (FOX), Cefotaxime (CTX), Cefepime (FEP)

RETRACTED

**Table 3:** Antibiotic resistance pattern for Gram-negative bacteria.

Antibiotics	N.gonorrhoeae (n = 33)			Klebsiella spp (n = 97)			P. aeruginosa(n = 195)			A. baumannii (n = 121)		
	U	R	S	U	S	R	U	S	R	U	S	R
**AMK**	**+**	**-**	**-**	**-**	**56**	**41**	-	**84**	**111**	**-**	**21**	**100**
**AMP**	**+**	**-**	**-**	**-**	**49**	**48**	-	**72**	**123**	**-**	**8**	**113**
**CZO**	**+**	**-**	**-**	**-**	**65**	**32**	-	**74**	**121**	**-**	**76**	**45**
**FEP**	**-**	**23**	**10**	**-**	**86**	**11**	-	**130**	**65**	**-**	**98**	**23**
**FOX**	**-**	**12**	**21**	**-**	**-**	**-**	+	**-**	**-**	**+**	**-**	**-**
**CRO**	**-**	**8**	**25**	**-**	**74**	**23**	-	**119**	**76**	**-**	**107**	**14**
**CIP**	**+**	**-**	**-**	**-**	**65**	**32**	-	**119**	**76**	**-**	**65**	**56**
**CLI**	**+**	**-**	**-**	**+**	**61**	**36**	-	**138**	**57**	**-**	**56**	**65**
**DOX**	**+**	**-**	**-**	**-**	**54**	**43**	-	**108**	**87**	**-**	**76**	**45**
**ERY**	**+**	**-**	**-**	**+**	**54**	**43**	-	**128**	**67**	**-**	**75**	**46**
**GEN**	**+**	**-**	**-**	**-**	**64**	**33**	-	**108**	**87**	**-**	**78**	**43**
**IMP**	**+**	**-**	**-**	**-**	**65**	**32**	-	**100**	**95**	**-**	**65**	**56**
**NIT**	**+**	**-**	**-**	**-**	**62**	**35**	-	**119**	**76**	**-**	**98**	**23**
**PEN**	**+**	**-**	**-**	**+**	**30**	**67**	-	**151**	**44**	**-**	**76**	**45**
**TZP**	**+**	**-**	**-**	**+**	**74**	**23**	-	**150**	**45**	**-**	**86**	**35**
**RIF**	**+**	**-**	**-**	**+**	**80**	**17**	-	**130**	**65**	**-**	**86**	**35**
**TCY**	**_**	**14**	**19**	**-**	**64**	**33**	-	**119**	**76**	**-**	**45**	**76**
**SXT**	**+**	**-**	**-**	**-**	**85**	**12**	-	**139**	**56**	**-**	**65**	**56**
**CAZ**	**_**	**21**	**12**	**-**	**54**	**43**	-	**138**	**55**	**-**	**65**	**56**
**SAM**	**+**	**-**	**-**	**+**	**52**	**45**	-	**150**	**45**	**-**	**76**	**45**
**LEV**	**+**	**-**	**-**	**-**	**74**	**23**	-	**150**	**45**	**-**	**56**	**65**
**MUP**	**+**	**-**	**-**	**+**	**-**	**-**	+	**-**	**-**	**+**	**-**	**-**
**MNO**	**+**	**-**	**-**	**+**	**63**	**34**	-	**139**	**56**	**-**	**56**	**65**
**LNZ**	**+**	**-**	**-**	**+**	**-**	**-**	+	**-**	**-**	**+**	**-**	**-**
**COL**	**+**	**-**	**-**	**-**	**85**	**12**		**177**	**18**		**100**	**21**
**CCV**	**+**	**-**	**-**	**+**	**82**	**15**	-	**172**	**23**	**-**	**97**	**25**

Abbreviations: Ampicillin (AMP), Gentamicin (GEN), Ciprofloxacin (CIP), Ceftazidime(CAZ), Nitrofurantoin (NIT), Imipenem (IMI), Penicillin (PEN), Clindamycin (CLI), Erythromycin (ERY), Doxycycline (DOX), Trimethoprim/sulfamethoxazole (SXT), Colistin (COL), Linezolid (LNZ), Mupirocin (MUP), Rifampin (RIF), Amikacin (AMK), Ceftriaxone (CRO), Ceftazidime/Clavulanic acid (CCV), Minocycline (MNO), Cefazolin (CZO), Cefepime (FEP), Piperacillin /Tazobactam (TZP), Tetracycline (TCY), Ampicillin/Sulbactam (SAM), Levofloxacin (LEV)

RETRACTED

### Antimicrobials resistant rates of (GPB) isolates from endotracheal tube cultures of patients

Table 2 depicts the prevalence of antibiotic resistance of GPB isolates. In case of *S*. *aureus* isolates, the highest resistance rates belonged to amikacin (n = 69/119; 57%), followed by penicillin (n = 64/119; 53%). However, *S*. *aureus* had no levels resistance to cefepime and Cefotaxime. In case of *Corynebacterium* spp and CoNS isolates, linezolid was the most efficient antimicrobials against. CoNS strains showed high-level resistance to levofloxacin (n = 88/100; 88%) and Ampicillin (n = 85/100; 85%). The percentage distribution rates of methicillin-resistant *Staphylococcus aureus* (MRSA) and methicillin-resistant CoNS (MR-CoNS) were 35% (n = 42/119) and 48% (n = 48/100), respectively. *Corynebacterium* spp. were 80% and 68% resistant to amikacin and cefepime, However, *Corynebacterium* spp. had low levels of resistance to linezolid and clindamycin. In case of *Streptococcus* spp. isolates, the highest resistance rates belonged to cefepime (n = 69/277; 65%), followed by penicillin (n = 64/277; 94%), clindamycin (n = 64/277; 59%) and tetracycline (n = 64/277; 68%). However, *Streptococcus* spp. had the low levels of resistance to rifampin and Trimethoprim-sulfamethoxazole. Detailed information on other GPBs is listed in Table 2.

### Antimicrobials resistant rates of (GNB) isolates from endotracheal tube cultures of patients

Among GNBs, *P*. *aeruginosa* isolates were 66% resistant to cefepime and 76% to colistin. However, *P*. *aeruginosa* showed low level of resistance to piperacillin /tazobactam and gentamycin. Colistin was the most effective antibiotic against *A*. *baumannii* and *Klebsiella* spp. *Klebsiella* spp isolates were resistant to ciprofloxacin in 71% of cases and amikacin in 67% of cases. Table 3 shows the incidences of resistance of each GNB to routinely used antimicrobials.

### Prevalence of MDR and XDR in GPB and GNB

The incidence rate of MDR and XDR bacterial infection from patients’ endotracheal tubes was determined by reference and is displayed in (Table 4) Out of total of 1136 bacterial strains studied, 365 (32%) bacterial strains were MDR, 441 (38%) strains were non- MDR, and 332 (29%) strains were XDR. Amongst 593 GPB strains isolated, 220 (37%) strains were MDR, 276 (46%) were non-MDR and 161(27.8%) XDR, respectively. Out from 546 GNB isolates, 146 (26%) were MDR, 276 (50%) were non-MDR, and 171 (31% were XDR). There was no evidence of a PDR strain. Table 4 illustrates the frequency of MDR and XDR rates of GNB and GNB.

RETRACTED

**Table 4:** Determination of MDR, NonMDR and XDR in bacterial isolates.

	MDR%	NonMDR%	XDR%
**Gram negative bacteria**			
*Acinetobacter spp(n = 121)*	94(77%)	15(12%)	12(0.09)
*Klebsiella spp*.*(n = 197)*	73(37%)	67(34%)	57(28%)
*P*. *aeruginosa (n = 195)*	43(22%)	75(38%)	77(39%)
*N*.*gonorrhoeae (n = 33)*	10(30%)	8 (24%)	15(45%)
Gram positive bacteria			
*S*. *aureus (n = 119)*	32(26%)	26(21%)	61(51%)
*Streptococcus spp*.*(n = 277)*	65(23%)	162(58%)	52(18%)
*CoNS (n = 100)*	23(23%)	44(44%)	33(33%)
*Enterococcus spp*.*(n = 32)*	13(40%)	6(18%)	13(40%)
*Corynebacterium*.*spp (n = 62)*	12(20%)	38(61%)	12(19%)

### Biofilm formation rates of GPB

Table 5 presents the data of biofilm formation using the MTP approach. Overall, of the 593 isolated bacteria, 429 (72%) were biofilm producers, of which, 292 (68%) produced strong biofilms, 83 (16%),292 (49%) produced moderate biofilms, 54 (12%) were weak biofilm producers and 221 (53%) were not biofilm producers. The capacity of biofilm formation in GPB are represented in Table 5.

**Table 5:** Biofilm formation of Gram-positive bacteria and Gram negative bacteria.

	Strong	Moderate	Weak	Non biofilm formation
Gram negative bacteria				
*Acinetobacter spp(n = 121)*	65(0.09)	12(0.09)	12(0.09)	32(0.09)
*Klebsiella spp*.*(n = 197)*	52(0.09)	34(0.09)	43(0.09)	68(0.09)
*P*. *aeruginosa(n = 195)*	49(0.09)	21(0.09)	29(0.09)	102(0.09)
*N*.*gonorrhoeae(n = 33)*	12(0.09)	6(0.09)	10(0.09)	5(0.09)
Gram positive bacteria				
*S*. *aureus(n = 119)*	64(0.09)	23(0.09)	2(0.09)	30(0.09)
*Streptococcus spp*.*(n = 277)*	144(0.09)	32(0.09)	13(0.09)	88(0.09)
*CoNS(n = 100)*	53(0.09)	10(0.09)	11(0.09)	86(0.09)
*Enterococcus spp*.*(n = 32)*	10(0.09)	5(0.09)	-	17(0.09)
*Corynebacterium*.*spp (n = 62)*	21(0.09)	13 (0.09)	28(0.09)	-

### Biofilm formation rates of GNB

The findings of biofilm formation using the MTP method are shown Table 5. In all, 345 (64.5%) of the 546 isolated bacteria were biofilm producers, with 178 (51%) formed strong biofilms, 73 (21%) generated moderate biofilms, 94 (27%) created weak biofilms, and 207 (6%) not developed biofilms. Table 5 illustrates the ability of GPB for biofilm development.

## Discussion

Following mechanical ventilation, VAP remains the most common problem, with a frequency rate of 3% during the first 5 days of ventilation, 2% between days 5 and 10, and 1% thereafter [19]. Identifying the resistance pattern of microorganisms, especially in every hospital, is an effective and acceptable technique for the treatment of VAP patients. In our hospital, the infections with Gram-positive (GPB) and Gram-negative (GNB) bacteria were 40% and 51%, respectively. Based on the results from the present study, VAP was greatly prevalent in ICU patients, and the majority of the GPB showed very high antibiotic resistance. Similarly, Lemmen et al. have reported GPB as the most frequent microorganisms isolated from the ET culture [20]. In our study, *Streptococcus* spp. was the most isolated GPB, and all of these microorganisms, regardless of S. aureus and *Enterococcus* spp., indicated 100% sensitivity to linezolid.

RETRACTED

In ICUs, a link has been found between MRSA and poor clinical outcomes, exerting a remarkable burden on infection control practices in hospitals. Likewise, the ICU is a critical place for the extensive spread of MRSA because patients are admitted and discharged to various wards and hospitals [21]. In this research, the prevalence of MRSA and CoNS were 35% and 48%, respectively. However, in another research made in Iran, the incidence of MRSA was found to be 72% [22], which is significantly greater than the proportion reported in the current study. In India, methicillin resistance of S. aureus infections has been reported to be 13–47% [21]. Patients in a (particularly surgical) ICU have wounds, drains, and invasive monitoring devices that result in skin breaches, thereby raising the risk of developing infections. Furthermore, because of the conditions such as diabetes, chronic liver disease, or steroid therapy, impaired neutrophil properties may cause the susceptibility of these patients to MRSA.

Among GNB, *Acinetobacter*, showed a high prevalence and multidrug resistance. Colistin was the only antibiotic that could relatively control the growth of the bacterium. Besides, the incidence of pneumonia or other infection caused by *Acinetobacter* was observed to be high. This observation is comparable with previous investigations in the ICUs [23, 24]. One study reported a high incidence of VAP, and *Citrobacter* and *Klebsiella* spp were the most prevalent organisms. The two bacteria were extremely resistant to carbapenems, a routinely used antibiotic in the ICU, but showed great sensitivity to colistin (94%) [25]. *Acinetobacter*, *Klebsiella*, and *Pseudomonas* were also highly resistant to GNB to third-generation cephalosporins and fluoroquinolones (> 80%). High resistance rates were recorded for aminoglycosides (> 68%) and imipenem (> 60%), whereas *Pseudomonas* resistance to piperacillin-tazobactam was lower than *Klebsiella* and *Acinetobacter* [26]. Other GNBs represented varied resistance patterns to the remaining antibiotics. Upadhyay and colleagues supported our finding and implied that *K*. *pneumoniae* was the main causative agent of VAP and resistant to third-generation antibiotics, cephalosporins, and penicillin. In contrast to the outcomes of both studies, the bacterium showed sensitivity to both carbapenems and polymyxin B [27]. Malik et al. have identified *K*. *pneumonia* as the most prevalent organism responsible for VAP and reported > 60% sensitivity of bacteria to combination drugs, i.e. Cefeperazone-sulbactam and Piperacillin-tazobactam [28]. Nevertheless, there are significant differences in the types of prevalent microorganisms, as well as antibiotic resistance and sensitivity, amongst all of the research described above. Considering these discrepancies, it is necessary for hospitals to continuously investigate the incidence of VAP-causing agents and to detect their antibiotic susceptibility by relying on available medications. The current investigation found a considerable number of MDR, which is consistent with previous findings of a high volume of multi-drug resistance [29–31]. The alarming rates of MDR and XDR in hospitals are indications of the fact that antibiotic resistance is raising, and pathogenic bacteria circulating in hospitals are obtaining high resistance to the majority of available antibiotics. In Iran, antibiotics can readily be purchased from pharmacies and private drug vendors without any prescription [32]. The existence of high rates of MDR and XDR will certainly enhance the rate of mortality in patients [33]. In the current study, most of our bacteria isolated were able to produce biofilm though with varied capacities. In organisms producing biofilms, there are different mechanisms, e.g. the weak diffusion of the antimicrobial penetration through the biofilm extracellular matrix, the various growth rate of biofilm organisms, and so on, that are responsible for antimicrobial resistance. Therefore, the ability to form biofilms may be a useful approach to enhance survival and persistence under stressful situations, such as host invasion or antibiotic treatment [34, 35].

RETRACTED

The present study explored that the capacity of biofilm formation has a significant correlation with antibiotic resistance (P<0.001). In other words, the density of biofilm in resistance strains was greater than in susceptible ones. In this regard, some researchers affirmed our study and displayed that the resistant isolates, compared to susceptible ones, were stronger biofilm producers [36, 37]. Overall, evaluating and comparing biofilm formation between non-MDR and MDR/XDR reflected that most of the MDR/XDR isolates possess a considerably higher capacity for the formation of biofilms in comparison to non-MDR isolates. As the biofilm dynamics are temporal, the development of VAP within the first 2–5 days following intubation is more likely to be caused by antibiotic-sensitive bacteria, namely methicillin-sensitive Staphylococcus aureus., with a better prognosis, later occurring VAP (5 or more days after initiation of mechanical ventilation) involving frequently multidrug-resistant pathogen like MRSA, P. aeruginosa and extended-spectrum β-lactamase producing Enterobacteriaceae, with higher morbidity and mortality [9]. Gordon Sahuquillo and co-workers examined the use of systemic and inhaled antibiotics on a small sample of patients and observed that the aforesaid antibiotics had no effect on the persistence of variables and potentially infectious microorganisms in ET biofilm after VAP. This resistance denotes the need for device withdrawal to attain microbiological and clinical cures; however, selective ET alteration during mechanical ventilation is often not recommended [38]. Within hours following insertion, the ET is quickly colonized by microorganisms forming a biofilm on its surface. Using scanning electron microscopy, Yan et al. evaluated biofilms formed on the surface of ET after initiating ventilation for 2–7 days and observed that biofilms covered a high percentage (87.5%) of ETs after 7–10 days. The last day (10th day) was the breakpoint when all the ETs housed biofilms on their surfaces. Indeed, the colonization of ET happens much earlier, though the validation of this matter is highly dependent on the methods assessed [1]. In a survey conducted by Adair and colleagues, in 70% of VAP patients, identical pathogens were found to exist in not only the ET biofilm but also in the lung, which is suggestive of the fact that the biofilm is an important and persistent source of pathogenic bacteria [39]. Future work with bigger populations may contribute to a deeper understanding of the microorganisms associated with the biofilm and their origins, as well as a clearer picture of the timing of biofilm formation and preventive treatments.

## Conclusions

The results of this study show that there is a large volume of microbial contamination in VAP, which can be very worrying, as well as instant antibiotic resistance on the surface. Considering the previous ability to pay attention to the formation of biofilm, it can place the need in the prescription of antibiotics to check the formation of biofilm in the practice of the hospital. Colistin and linezolid are effective antibiotics against practically all resistant GPB and GPB isolates, but the elevated level of their innate resistance to antibacterial often results in the emergence of Gram-positive and gram negative bacteria. Hence, excessive use of these medications should be approached with extreme caution.

RETRACTED

## List of abbreviations

VAP: ventilator-associated pneumonia
GPB: Gram-negative bacteria
GPB: Gram-positive bacteria
ET: Endotracheal tube
MDR: Multiple drug resistance
XDR: Extensively drug-resistant
PDR: Pan drug-resistant
MTP: Microliter Plate
MRSA: Methicillin-resistant Staphylococcus aureus
CoNS: Coagulase-negative staphylococci
MR-CoNS: Methicillin-resistant Coagulase-negative staphylococci
TSB: tryptic soy broth
DM: diabetes mellitus
HTN: : hypertension
OD: Optical Density
MIC: minimum inhibitory concentration
CLSI: Clinical & Laboratory Standards Institute
ICU: Intensive care units
